The article "LacI-Family Transcriptional Regulator DagR Acts as a Repressor of the Agarolytic Pathway Genes in Streptomyces coelicolor A3(2)" was retracted in 2022. Reasons: fabricated or falsified data; fabricated or falsified images.

# LacI-Family Transcriptional Regulator DagR Acts as a Repressor of the Agarolytic Pathway Genes in *Streptomyces coelicolor* A3(2)

**DOI:** 10.3389/fmicb.2021.658657

**Published:** 2021-04-06

**Authors:** Maral Tsevelkhoroloo, So Heon Shim, Chang-Ro Lee, Soon-Kwang Hong, Young-Soo Hong

**Affiliations:** ^1^Department of Bioscience and Bioinformatics, Myong-Ji University, Yongin-si, South Korea; ^2^Anticancer Agent Research Center, Korea Research Institute of Bioscience and Biotechnology, Cheongju-si, South Korea

**Keywords:** *Streptomyces coelicolor* A3(2), repressor, agarolytic pathway, LacI-family transcriptional regulator, DagR represses agarase genes in *S. coelicolor*

## Abstract

Actinobacteria utilize various polysaccharides in the soil as carbon source by degrading them via extracellular hydrolytic enzymes. Agarose, a marine algal polysaccharide composed of D-galactose and 3,6-anhydro-L-galactose (AHG), is one of the carbon sources used by *S. coelicolor* A3(2). However, little is known about agar hydrolysis in *S. coelicolor* A3(2), except that the regulation of agar hydrolysis metabolism is strongly inhibited by glucose as in the catabolic pathways of other polysaccharides. In this study, we elucidated the role of DagR in regulating the expression of three agarase genes (*dagA*, *dagB*, and *dagC*) in *S. coelicolor* A3(2) by developing a *dagR*-deletion mutant (Δsco3485). We observed that the Δsco3485 mutant had increased mRNA level of the agarolytic pathway genes and 1.3-folds higher agarase production than the wild type strain, indicating that the *dagR* gene encodes a cluster-suited repressor. Electrophoretic mobility shift assay revealed that DagR bound to the upstream regions of the three agarase genes. DNase 1 footprinting analysis demonstrated that a palindromic sequence present in the upstream region of the three agarase genes was essential for DagR-binding. Uniquely, the DNA-binding activity of DagR was inhibited by AHG, one of the final degradation products of agarose. AHG-induced agarase production was not observed in the Δsco3485 mutant, as opposed to that in the wild type strain. Therefore, DagR acts as a repressor that binds to the promoter region of the agarase genes, inhibits gene expression at the transcriptional level, and is derepressed by AHG. This is the first report on the regulation of gene expression regarding agar metabolism in *S. coelicolor* A3(2).

## Introduction

*Streptomyces* sp. is one of the most important sources of bioactive secondary metabolites. Its capability of utilizing various insoluble polysaccharides present in the soil has evolved due to the production of various extracellular hydrolytic enzymes, such as protease, chitinase, cellulase, amylase, and xylanase, and in rare cases, agarase (Kim et al., 2008; Chater et al., 2010).*Streptomyces coelicolor* A3(2), a model organism of this genus, is the only species that has the unusual capability of utilizing agar as the sole carbon source (Kendall and Cullum, 1984). Genomic sequencing of *S. coelicolor* A3(2) has shown that there are at least 819 predicted secretion proteins (Bentley et al., 2002), some of which assist in the digestion of the nutrients present in the soil; it includes a gene cluster, which is involved in agar degradation (Hsiao and Kirby, 2008). Although the *S. coelicolor* A3(2) agarolytic pathway has not been widely studied, the first secretory β-agarase (DagA; coded by *sco3471*) was identified to degrade agarose into neoagarotetraose and neoagarohexaose (Bibb et al., 1987; Buttner et al., 1987, 1988; Temuujin et al., 2011; Park et al., 2014). In a previous study, we reported DagB (coded by *sco3487*), an exo- and endo-type β-agarase that degrades agarose, neoagarotetraose, and neoagarohexaose into neoagarobiose as the major product. DagA and DagB work together enhance the hydrolysis of agarose into neoagarobiose (Temuujin et al., 2012). In addition, we proposed that neoagarobiose could be transported into the cytosol by a transporter protein and hydrolyzed into the constituent monomers D-galactose and 3,6-anhydro-L-galactose (AHG) by DagC (coded by *sco3481*) (Chi et al., 2012).

The article "LacI-Family Transcriptional Regulator DagR Acts as a Repressor of the Agarolytic Pathway Genes in Streptomyces coelicolor A3(2)" was retracted in 2022. Reasons: fabricated or falsified data; fabricated or falsified images.

Genetic studies on the agarolytic pathway have identified that glucose strongly represses the transcription of *dagA*, which is transcribed from four promoters that are recognized by probably four different RNA polymerase holoenzymes, each containing a different σ factor (Buttner et al., 1987, 1988; Servin-Gonzalez et al., 1994). As expected, the other agarase genes (*dagB* and *dagC*) are also repressed by glucose (Romero-Rodriguez et al., 2016). This glucose catabolite repression was observed in a large genomic region (*sco3471*-*sco3487*), which contains the three agarase genes. However, DagR (coded by *sco3485*), a putative LacI-family transcriptional regulator, was not repressed by glucose although it was the only regulator in this cluster (Chi et al., 2012; Romero-Rodriguez et al., 2016, 2017).

LacI-family transcriptional regulators are a group of allosteric DNA-binding regulators with conserved amino acid sequences (Lewis, 2005). Majority of the characterized LacI-family transcriptional regulators sense sugar effectors and regulate carbohydrate utilization genes (Ravcheev et al., 2014). In bacteria, the lactose repressor LacI of *Escherichia coli* has been used as the model for the analysis of bacterial transcriptional regulation. In this study, we elucidated the role of DagR in regulating the expression of *dagA*, *dagB*, and *dagC* in *S. coelicolor* A3(2) by developing a *dagR* deletion mutant (Δsco3485). We demonstrated that the Δsco3485 mutant strain had increased agar degradation activity compared with that of the wild type *S. coelicolor* A3(2) and that DagR deficiency strongly induced the transcriptional level of agar hydrolytic genes. Additionally, we validated that DagR bound *in vitro* to consensus palindromic sequences located upstream of the three agarase genes. In addition, the binding activity of DagR was inhibited by AHG. AHG increased the agarase activity in *S. coelicolor* A3(2) strain but was not effective in the Δsco3485 mutant. All these results and phenotypic analyses clearly demonstrated that DagR acts as a transcriptional repressor of the agarolytic pathway in *S. coelicolor* A3(2), which is the first report on regulation of gene expression regarding agar metabolism.

The article "LacI-Family Transcriptional Regulator DagR Acts as a Repressor of the Agarolytic Pathway Genes in Streptomyces coelicolor A3(2)" was retracted in 2022. Reasons: fabricated or falsified data; fabricated or falsified images.

## Materials and Methods

### Bacterial Strains and Culture Conditions

All bacterial strains and plasmids used in this work are summarized in Table 1. The *E. coli* strain was grown in *Luria–Bertani* (LB) broth. The media and manipulation techniques required for culturing *Streptomyces* are described in the *Streptomyces* manual (Kieser et al., 2000). If necessary, antibiotics were added to the medium as follows: apramycin (50 μg/mL), chloramphenicol (25 μg/mL), kanamycin (50 μg/mL), thiostrepton (50 μg/mL), and nalidic acid (25 μg/mL). Primers are listed in Supplementary Table 1.

**TABLE 1:** Bacterial strains and plasmids used in this work.

Plasmid or strain	Description	Source or references
pET-28a(+)	f1 *ori*, T7 promoter, Kan^R^	Novagen
pET-3485	pET-28a(+) carrying *dagR* (*sco3485*) gene from *S. coelicolor*	This study
pWHM3	*E. coli*-*Streptomyces* shuttle vector, Tsr^*R*^, Amp^*R*^	Kieser et al., 2000
pWHM-3485	Complementation plasmid, pWHM3 carrying *dagR* gene	This study
pCRISPomyces-2	Streptomyces CRISP/cas9 vector, Apr^*R*^, *oriT*, *rep^pSG5(ts)^*, *ori^ColE1^*, *sSpcas9*, synthetic guide RNA cassette	Cobb et al., 2015
dCRI-3485	pCRISPomyces-2 with *dagR* sgRNA and 2kb editing template	This study
*Streptomyces coelicolor* A3(2)	Agarases producer; SCP1^–^, SCP2^–^	Kieser et al., 2000
Δsco3485	*S. coelicolor* A3(2) with 64-bp deletion on *dagR* gene	This study
Δsco3485/pWHM-3485	Δsco3485 carrying pWHM-3485	This study
*E. coli* DH5α	Cloning host	Invitrogen
*E. coli* BL21(DE3)	Protein overexpression strain	Novagen
*E. coli* BL21(DE3)/pET-3485	*E. coli* BL21(DE3) carrying pET-3485	This study
*E. coli* ET12567	RP4-Tc::Mu-Km::Tn7, Cm^*R*^ *dam*^–^, *dcm*^–^, *hsdM*^–^	Kieser et al., 2000
*E. coli* ET12567/pUZ8002	ET12567 carrying pUZ8002 (*oriT* mobilizing plasmid, Km^R^)	Kieser et al., 2000

**Amp^*R*^, ampicillin; Apr^*R*^, apramycin; Km^*R*^, kanamycin; Cm^*R*^, chloramphenicol; Tet^*R*^, tetracycline; Tsr^*R*^, thiostrepton.**

The article "LacI-Family Transcriptional Regulator DagR Acts as a Repressor of the Agarolytic Pathway Genes in Streptomyces coelicolor A3(2)" was retracted in 2022. Reasons: fabricated or falsified data; fabricated or falsified images.

### DNA Manipulation and Plasmid Construction

All DNA manipulations were performed according to the standard procedures for *E. coli* and *Streptomyces* (Sambrook et al., 1989; Kieser et al., 2000). All kits and enzymes were used according to the manufacturer’s recommendations. For the expression of DagR in *E. coli*, a 1,089-bp fragment (the entire coding sequence of *dagR*) was amplified by PCR using the primers (SCO3485-F and R), and then inserted into the *Nde*I and *Hin*dIII sites of pET-28a, yielding pET-3485. For the expression of DagR in *Streptomyces*, a 1,415-bp fragment (including the promoter and coding sequence of *dagR*) was amplified by PCR using the primers (SCO3485com-F and R), and then ligated into the *Eco*RI and *Hin*dIII sites of pWHM3, yielding pWHM-3485. The CRISPR-Cas9 deletion system for *dagR* gene was constructed based on pCRISPomyces-2 (Cobb et al., 2015), and the single synthetic guide RNA sequence with the nearby protospacer adjacent motif (PAM) sequence was analyzed using BLAST to confirm its specificity. The 20-bp sequence with the requisite PAM sequence was synthesized (sgRNA-3485F and sgRNA-3485R) and inserted into pCRISPomyces-2 plasmid through Golden Gate assembly (Cobb et al., 2015). Next, two approximately 1-kb homologous arms corresponding to the upstream and downstream regions of the target gene (*dagR*) were amplified from purified genomic DNA and fused into the *Xba*I site of the desired deletion plasmid (dCRI-3485).

### Construction and Complementation of Δsco3485 Mutant

Plasmid dCRI-3485 is a derivative of pCRISPomyces-2 for targeted *dagR* gene deletions in *S. coelicolor* A3(2). The plasmid was delivered into *S. coelicolor* A3(2) by intergeneric conjugation according to standard procedures using *E. coli* ET12567(pUZ8002) (Kieser et al., 2000). Following conjugation, individual exconjugants were randomly picked and restreaked on R2YE agar plates supplemented with 50 μg/mL apramycin and grown at 28°C for 2–3 days. Clearance of the temperature-sensitive plasmid was accomplished with high-temperature cultivation (40°C) for 2–5 days, followed by replica plating on selective and non-selective plates to confirm loss of apramycin resistance. To determine the CRISPR-Cas9 mediated recombination, each selected apramycin sensitive colony was subjected to PCR using the primers (C3485-F and C3485-R). The locus of interest was PCR amplified and sequenced using primers annealing 46-bp upstream and downstream of the deletion site. Thus, a ∼400-bp fragment was expected from the mutant strain (Δsco3485) in contrast to the 464-bp fragment expected from the wild type strain (Supplementary Figure 1). To complement the Δsco3485 mutant, a recombinant vector pWHM-3485 containing the *dagR* gene was isolated from *E. coli* ET12567, which was transformed into the Δsco3485 mutant again by PEG transformation protocol (Kieser et al., 2000). The transformant *S. coelicolor* Δsco3485/pWHM-3485 was cultured and maintained in the presence of thiostrepton (50 μg/mL).

The article "LacI-Family Transcriptional Regulator DagR Acts as a Repressor of the Agarolytic Pathway Genes in Streptomyces coelicolor A3(2)" was retracted in 2022. Reasons: fabricated or falsified data; fabricated or falsified images.

### Analysis of Agarase Activity by Zymogram Assay and Dinitrosalicylic Acid (DNS) Method

For zymogram analysis, each strain was spotted onto a R2YE agar plate and grown at 2–7 days. The plates were then stained with Lugol’s iodine solution (25 g of iodine and 50 g of potassium iodine in 1 L of distilled water) at room temperature. The agarase activity of the liquid culture was quantified using the DNS method (Temuujin et al., 2011). Each strain was inoculated into modified RSM3 (glucose 25 g, MgCl_2_ 6H_2_O 5 g, yeast extract 11 g, CaCO_3_ 2 g, per L) broth to which 0.2% acidified agar (AO) was added, and cultured at 28°C for 7 days. During cultivation, 1 mL was sampled and the cells and the supernatant were separated by centrifugation (10,000 × g, 20 min, 4°C). To measure the agarase activity of the supernatant, 10 μL of the culture solution was mixed with 490 μL of 50 mM sodium phosphate buffer (pH 7.0) containing 0.2% agarose. After reacting at 40°C for 10 min, the mixture was mixed with 500 μL of DNS reagent solution (DNS 6.5 g, 2 M NaOH 325 mL, glycerol 45 mL in 1 L of distilled water) and heat treated for 10 min in boiling water. The reaction solution was cooled in an ice bath, and the absorbance at 540 nm (A_540_) was measured with a UV spectrometer. As a blank, a culture solution heat-treated for 10 min was used. The dry weight of the cells was measured after the centrifuged pellet was washed twice by centrifugation with 50 mM sodium phosphate buffer (pH 7.0), dried at 40°C for 24 h. The data shown in this study were generated from triplicate independent experiments.

### RNA Extraction and RNA-Seq Analysis

For RNA preparation, the fresh spores of wild type *S. coelicolor* and Δsco3485 strain were inoculated into 250-mL Erlenmeyer flasks containing 25-mL liquid R2YE and incubated at 28°C for 48 h. The seed cultures were inoculated in liquid modified RSM3 medium with a dilution ratio of 1:20, and cultivated for 4 days at 28°C. The cultured cell pellets (seeding cells as control and 4-day cultured cells) were quickly harvested, flash frozen in liquid nitrogen, and then ground into powder. Total RNA was purified using RNeasy Mini kit (Qiagen, Germany) according to the manufacturer’s instructions. The total RNA of *S. coelicolor* A3(2) and Δsco3485 strain samples was used for massively parallel cDNA sequencing to present a genome-wide map of transcript levels. Details of the RNA-Seq was carried out in accordance with the manufacturer’s protocol (BGI Tech Solutions, Shenzhen, China). Clean reads of each sample were mapped with NCBI *S. coelicolor* A3(2) reference genome (Bentley et al., 2002) using Tophat2 to obtain BAM file. BAM files were sorted, indexed with Samtools, and the FPKM was calculated with Cufflinks (v2.2.1). With FPKM values, differentially expressed genes (DEGs) and statistical analysis was performed. Fold-change values were calculated by dividing FPKM of control and that of treated sample. >2 × fold-changed value between control and treated sample was considered as differentially expressed.

The article "LacI-Family Transcriptional Regulator DagR Acts as a Repressor of the Agarolytic Pathway Genes in Streptomyces coelicolor A3(2)" was retracted in 2022. Reasons: fabricated or falsified data; fabricated or falsified images.

### Purification of the His-Tagged DagR Protein Expressed in *E. coli*

*E. coli* BL21(DE3) cells transformed with pET-3485 were inoculated in 100 mL of LB medium added with kanamycin and cultured at 37°C. When the optical density (OD_600_) of the culture broth measured at 600 nm was 0.6, isopropyl-D-thiogalactopyranoside (IPTG, 0.5 mM) was added to induce DagR expression. After culturing for 16 h under the same conditions, the cells were harvested by centrifugation (10,000 × g, 20 min, 4°C). The cell-free lysate was obtained by centrifugation (15,000 × g, 30 min, 4°C) of the total cell lysate prepared by sonication, which was used for purification of the His-tagged DagR protein by using a BD TALON^TM^ metal affinity resin (Clontech Laboratories Inc., United States). The purified His-tagged DagR protein (Supplementary Figure 3) was used for electrophoretic mobility shift analysis (EMSA) and DNase 1 footprinting.

### Electrophoretic Mobility Shift Assay (EMSA)

The promoter regions of *dagA* (371 bp), *dagB* (390 bp), *dagC* (284 bp) genes were amplified from *S. coelicolor* A3(2) genomic DNA by PCR with each biotin labeled primer set (Supplementary Table 1). EMSAs were performed with approximately 1 nM biotin-labeled DNA probe and excess of non-specific competitor DNA. Binding reactions were prepared in binding buffer (20 mM Tris-HCl (pH 8.0), 1 mM MgCl_2_, 0.1 mM dithiothreitol (DTT), 12.5% glycerol, 50 mM NaCl, 0.4 mM EDTA) at 28°C for 20 min. Each 20-μL binding reaction mixture, containing the biotinylated DNA probe at 1 nM and the purified His-tagged DagR protein at various concentrations (0–19.1 μM). After binding, the mixture was separated on 5% TBE gel, buffered in 0.5 × TBE buffer at 100 v, and bands were detected by BeyoECL Plus (Thermo Fisher Scientific). The unlabeled probe (cold) was used as a competitor. EMSA was performed on agarose gel electrophoresis (1.2% agarose gel in TBE buffer) instead of PAGE to investigate the effect of various sugars on 19.1 μM (15 μg) of DagR binding. D-Glucose, D-galactose, neoagarobiose, agarotriose, and agaropentaose mixture (A3 + A5), neoagarotetraose and neoagarohexaose mixture (NA4 + NA6), and 3,6-anhydro-L-galactose (AHG) were added at various concentrations (0, 15, 20, and 30 μg) into EMSA reaction separately. Neoagarobiose, agarotriose and A3 + A5 mixture, and NA4 + NA6 mixture were purchased from Dynebio Inc. (Seongnam, South Korea), and AHG was prepared by enzymatic digestion of agarose with an agarase mixture (purified DagA, DagB, and DagC enzymes) as previously reported (Temuujin et al., 2011, 2012).

The article "LacI-Family Transcriptional Regulator DagR Acts as a Repressor of the Agarolytic Pathway Genes in Streptomyces coelicolor A3(2)" was retracted in 2022. Reasons: fabricated or falsified data; fabricated or falsified images.

### Mapping of the DagR-Binding Sites by DNase 1 Footprinting

The DNase 1 footprinting analysis was carried out by capillary DNA sequencer using a fluorescent labelled PCR fragment as previously published (Yindeeyoungyeon and Schell, 2000). The primers used for each promoter region were labeled with 5′ 6-FAM on primers having the same sequence as those used in the previous EMSA experiment (Supplementary Table 1). The labeled DNA probes (540 ng) were incubated with the DagR protein (25 μg) at 28°C for 20 min in the binding buffer (20 mM Tris-HCl (pH 8.0), 1 mM MgCl_2_, 0.1 mM DTT, 12.5% glycerol, 50 mM NaCl, 0.4 mM EDTA). The digestion of DNA probe was performed at 37°C using 1 unit of DNase 1 (Promega) per 50 μL reaction solution. Five minutes after the reaction, a stop buffer (130 mM NaCl, 20 mM EDTA, 0.6% SDS) was added the reaction, and the digested DNA probe was purified with a PCR Purification kit (Qiagen). The fluorescence patterns of the sample were analyzed by using a 3730 automated DNA sequencer (Applied biosystems, United States) by the Macrogen (Seoul, South Korea). Electropherograms indicate the protected patterns of the each promoter after digestion with DNase 1 following incubation with DagR protein.

### Evaluation of Agarase Activity After Adding AHG

All the strains were cultivated in RSM3 broth (10 mL) at 28°C for 24 h. Then, AHG (10 mM) was added to each culture solution, and the samples (1 mL) were taken at intervals while culturing at 28°C. After centrifugation at 10,000 × g for 10 min, the supernatant (10 μL) was mixed with 490 μL of 50 mM sodium phosphate buffer (pH 7.0) containing 0.2% agar. The agarase activity was quantified by using the DNS method described above. The precipitate was used for measuring cell dry weight. The data shown in this study were generated from triplicate independent experiments.

The article "LacI-Family Transcriptional Regulator DagR Acts as a Repressor of the Agarolytic Pathway Genes in Streptomyces coelicolor A3(2)" was retracted in 2022. Reasons: fabricated or falsified data; fabricated or falsified images.

## Results

### *dagR* (*sco3485*), Encode a LacI-Family Transcriptional Regulator, Which Acts as a Repressor of the Agarolytic Pathway Genes in *S. coelicolor* A3(2)

In *S. coelicolor* A3(2), agarolytic pathway genes, including the three agarase genes, *dagA*, *dagB*, and *dag*C, are located in a cluster on the chromosome (Bentley et al., 2002; Figure 1). Each of the three genes is essential for agarose utilization in this bacterium. The *dagR* (*sco3485*) is the only putative regulatory gene found in the agarolytic pathway gene cluster. The DagR protein encoded by the ORF of *dagR* comprises 349 amino acids with a calculated molecular mass of 37 kDa. The N terminus of the protein is characterized by a helix–turn–helix motif, which is characteristic of the LacI-family (Nguyen and Saier, 1995), suggesting that DagR functions as a transcriptional regulator in carbohydrate utilization (Perez-Rueda and Collado-Vides, 2000).

**FIGURE 1:** **(A)** Genomic organization of the agarolytic pathway genes in *S. coelicolor* A3(2). **(B)** Schematic illustration of the DagR protein and sequence alignments of the N-terminal region of DagR homologs in which the fully conserved regions are indicated by a black background. The microorganisms of source and accession numbers are: LacI from *E. coli* (QCB65867); RbsR from *Serratia* (WP141971870); PurR from *S. coelicolor* (CAC10103); CebR from *Streptomyces* (WP003968984); MalR from *S. coelicolor* (P09371).

To assess any impacts on agarose utilization, mutation of the *dagR* gene was performed using the CRISPR-cas9 system (Cobb et al., 2015). The Δsco3485 mutant was found to have a 64-bp deletion at the 5′ end of the *dagR* gene (Supplementary Figure 1). The agarase activity of the Δsco3485 mutant showed a significant increase in both liquid medium and solid agar plates compared to that of the wild type *S. coelicolor* strain (Figure 2). The agarase activity of the Δsco3485 mutant increased from day 2 and reached its maximum level (A_540_ = 1.2 ± 0.03) after 5 days of growth in liquid medium. The Δsco3485 mutant showed 1.3-folds more agarase activity than the controls. The agarase activity of the Δsco3485 mutant reduced to the level of wild type strain in liquid medium after complementation with the *dagR* gene (Δsco3485/pWHM–3485). While there was no significant difference in the cell growth rate of both type of strains, enhanced agarase expression by the Δsco3485 mutant since early growth phase could be due to the deletion of the *dagR* gene.

**FIGURE 2:** Comparison of agarase activity of the wild type *S. coelicolor* A3(2) strain and the Δsco3485 mutant. Zymogram plate assay **(A)** results of the Δsco3485 mutant as a function of cultivation time. The cells were grown on R2YE agar plates for the indicated times and were stained with Lugol’s solution. Agarase production **(B)** and cell growth **(C)** as a function of cultivation time. Strains were grown at 28°C in RSM3 medium for 7 days and samples were collected to measure cell growth (g protein/liter) and agarase activity. All data shown are mean values from at least three replicate experiments. Error bars indicate standard deviations of the means (*n* = 3). Agarase activity and cell growth of the Δsco3485 mutant (◼), wild type *S. coelicolor* A3(2) (□), and complement strain (Δsco3485/pWHM-3485) (▲).

The article "LacI-Family Transcriptional Regulator DagR Acts as a Repressor of the Agarolytic Pathway Genes in Streptomyces coelicolor A3(2)" was retracted in 2022. Reasons: fabricated or falsified data; fabricated or falsified images.

To examine the relationship between agarase activity and transcriptomic changes, RNA sequencing (RNA-seq) analysis was conducted using 4-day old cultures grown in liquid modified RSM3 medium. RNA-seq detected that 8,299 coding genes were transcribed during growth of the wild type strain and the Δsco3485 mutant on the modified RSM3 medium for 4 days. To assess the differentially expressed genes (DEGs) in the wild type strain and Δsco3485 mutant, the criteria were set as fold change of >2.0 or <2.0 (*P* < 0.05). Among the 1,040 DEGs analyzed using the DESEQ package, 278 genes were up-regulated and 319 genes were down-regulated in the Δsco3485 mutant as compared to that in the wild type strain (Supplementary Tables 2, 3). All agarolytic pathway genes (*sco3471*-*3487*) were remarkably upregulated compared to other genes (Figure 3 and Supplementary Figure 2). Interestingly, it was confirmed that the expression of the three agarase genes, the genes assumed to be related to AHG metabolism, and the sugar transporter-associated gene (*sco3482*-*3484*), which exists in the central region of the agarolytic pathway gene cluster, were all significantly increased. Thus, same expression pattern for all of genes in this cluster could mean that they have a common regulator. All the genes in the cluster were over-expressed in the absence of intact DagR, which indicated that their expressions may be regulated by the regulator present in the cluster, DagR.

**FIGURE 3:** Heatmap of the expression of the agarolytic pathway genes (*sco3471*-*3487*) depicting fold-changes in the Δsco3485 mutant compared to the wild type strain. The cultured cell pellets [seeding cells as control (0-day) and 4-day cultured cells] were used for RNA purification.

### DagR Protein Binds to the Upstream Regions of *dagA*, *dagB*, and *dagC*

To confirm the ability of the DagR protein to bind to the upstream regions of the three agarase genes, electrophoretic mobility shift assay (EMSA) was performed using the His-tagged DagR protein, which was expressed in *E. coli* and purified (Supplementary Figure 3). A biotin-labeled DNA fragment containing the upstream regions of *dagA*, *dagB*, and *dagC* served as the binding partner in the EMSA studies. DNA fragments of 371 bp (pdagA; between positions –365 and +6 with respect to the *dagA* translation start site), 390 bp (pdagB; between positions –390 and –1 with respect to the *dagB* translation start site), and 284 bp (pdagC; between positions –311 and –27 with respect to the *dagC* translation start site) were used as DNA probes for *dagA*, *dagB*, and *dagC*, respectively (Figure 4). The DagR protein reduced the electrophoretic mobility of the all of three upstream DNA fragments; the amount of the DagR-DNA complex increased as the concentration of the DagR protein increased (Figure 4). EMSA results clearly revealed that the DagR protein bound to the upstream DNA fragments of *dagA*, *dagB*, and *dagC*. Interestingly, a complete band-shift with pdagA DNA fragment was achieved after addition of 2.5 μM DagR protein, but the band-shift with pdagB and pdagC DNA fragments was achieved after addition of 8.9 μM and 6.4 μM DagR protein, respectively. Although these results do not confirm that DagR protein preferred binding with pdagA DNA fragment over the other two DNA fragments, it is highly possible that each DNA fragment can have a different binding affinity for DagR protein.

The article "LacI-Family Transcriptional Regulator DagR Acts as a Repressor of the Agarolytic Pathway Genes in Streptomyces coelicolor A3(2)" was retracted in 2022. Reasons: fabricated or falsified data; fabricated or falsified images.

**FIGURE 4:** *In vitro* binding of DagR to the upstream regions of the three agarase genes, *dagA*, *dagB*, and *dagC*. EMSA was carried out with the purified His-tagged DagR protein. The DNA probes used were the upstream regions of *dagA* (pdagA) **(A)**, *dagB* (pdagB) **(B)**, and *dagC* (pdagC) **(C)**. Each 20-μL binding reaction mixture, containing the biotinylated DNA probe at 1 nM and the DagR protein at various concentrations (0–19.1 μM), was subjected to electrophoresis on a 6% polyacrylamide gel. Cold, unlabeled probe.

### Identification of DagR-Binding Sites in the Upstream Regions of *dagA*, *dagB*, and *dagC*

As a band-shift was achieved by the addition of DagR protein, we searched for the DagR-binding motif in the putative promoter region of the three agarase genes. We performed DNase 1 footprinting analysis to determine the DagR-binding sites within the promoter fragment region of *dagA*, *dagB*, and *dagC*. The promoter fragment was used by labeling the same fragment used in the previous EMSA experiment with a fluorescent dye. Electropherograms indicate the protected patterns of each promoter after digestion with DNase 1 following incubation with DagR protein (Figure 5). The results showed that the region of *dagA* promoter protected by DagR was –219 to –212 nt (5′- AACCGGTT-3′). Furthermore, the regions of *dagB* promoter protected by DagR were –111 to –102 nt (5′- AAACCGGTTT -3′) and –364 to –357 nt (5′- GGACGTCC -3′), whereas the region of *dagC* promoter protected by DagR was –179 to –172 nt (5′- CCGATCGG-3′) (Figure 5). The binding motifs of most LacI-family transcription regulators are palindromes formed by highly conserved inverted repeats (Ravcheev et al., 2014). In this study, the binding sequence in the upstream region of *dagA* and the first binding site of *dagB* showed the highly conserved inverted repeat (AACCGGTT), but the binding sequence in the upstream region of *dagC* (CCGATCGG) and the second binding site of *dagB* (GGACGTCC) were palindromes and not homologous. In particular, the conserved binding sequence (AACCGGTT) was located in the fourth of the four transcription start sites of *dagA* identified by Buttner et al.(1987; Figure 6).

The article "LacI-Family Transcriptional Regulator DagR Acts as a Repressor of the Agarolytic Pathway Genes in Streptomyces coelicolor A3(2)" was retracted in 2022. Reasons: fabricated or falsified data; fabricated or falsified images.

**FIGURE 5:** DNase 1 footprinting assays for the identification of DNA motif bound by DagR. Electropherograms showing the protection pattern of each promoter of fluorescent dye-labeled upstream region of *dagA* **(A)**, *dagB* **(B)**, and *dagC* **(C)** after digestion with DNase 1 following incubation in the absence (up) or presence (bottom) of DagR protein. The *y*-axis gives fluorescence intensity (i.e., fragment abundance), while the *x*-axis (upper) gives elution position, which is proportional to size. At the bottom is a scale that gives nucleotide position relative to the each gene. The protected regions are indicated with red box, and the palindrome sequences (DagR-binding sites) are shown below. The numbers refer to the distance from translation start site of the each gene.

**FIGURE 6:** Nucleotide sequence of the promoter regions of *dagA*. Sequences of DagR-binding sites are in bold and red. The transcription start sites of *dagA* are indicated by a circle and black arrow above the corresponding nucleotide. The putative -10 and -35 regions and the ribosomal binding sites (SD) are underlined and in green. The signal peptide sequence of DagA is underlined. The position of the PCR primers used for DNase 1 footprinting analysis is marked by a tangent arrow.

### DagR-Binding in the Upstream Regions of *dagA* Is Inhibited by AHG

The effects of various sugars on the DNA-binding activity of the DagR protein were examined by EMSA (Figure 7). Different amounts of sugars with DagR protein (15 μg) were incubated with the DNA fragment. D-Glucose, D-galactose, neoagarobiose, A3 + A5 mixture, NA4 + NA6 mixture, and AHG were added into EMSA reaction separately. The results showed that DagR could bind to the dagA promoter in the presence of glucose, galactose, neoagarobiose, and (neo)agaro-oligosaccharides mixtures (Figure 7). However, in the presence of AHG (15 μg), free DNA bands of the *dagA* promoter (pdagA) were observed although some DNA-protein complex band was present. At a concentration of 20 μg, AHG clearly reduced the formation of the complex of DagR with the *dagA* upstream DNA fragment. In contrast, other sugars did not affect the DNA-binding activity of DagR even at 30 μg. Thus, these results indicated that AHG inhibited the binding of DagR to the *dagA* promoter region. It is estimated that AHG, which is a product whose neoagarobiose has been digested by DagC enzymes (Chi et al., 2012), could activate the expression of the agarolytic pathway genes as a negative effector of the binding activity of DagR.

The article "LacI-Family Transcriptional Regulator DagR Acts as a Repressor of the Agarolytic Pathway Genes in Streptomyces coelicolor A3(2)" was retracted in 2022. Reasons: fabricated or falsified data; fabricated or falsified images.

**FIGURE 7:** Effects of various sugars on the DNA-binding activity of DagR. EMSA was carried out with the DagR protein and the *dagA* upstream region. Each 20-μL binding reaction mixture, containing the DNA probe pdagA (Figure 4) at a concentration of 15 μg (19.1 μM) with or without the DagR protein, was subjected to electrophoresis on an agarose gel. The reaction mixture was supplemented with sugars at various concentrations (0, 15, 20, and 30 μg). The free DNA and the DNA-protein complex are indicated by parentheses and black arrowheads, respectively.

### Induction of Agarase Production by AHG Is Dependent on DagR

Because AHG could suppress the DNA-binding activity of DagR, the phenotypic response of the Δsco3485 mutant and the wild type strain to AHG was compared (Figure 8). When AHG was added to the 24 h cultured broth, the wild type strain showed an increase in agarase production to the level of Δsco3485 mutant after 12 h, and maintained higher production than the culture without AHG till 24 h, indicating that AHG induced the expression of agarases. Consistent with the results shown in Figure 2, the Δsco3485 mutant had higher agarase production capacity than that of the wild type strain, but did not show induction of agarase expression by the addition of AHG. These results strongly imply that the induction of agarase expression by AHG is dependent on intact DagR, and therefore AHG induces agarase gene expression by inhibiting the ability of DagR to bind to the DNA target sites.

**FIGURE 8:** Change of agarase activity in the wild type strain and Δsco3485 mutant by the addition of AHG. All strains were grown at 28°C in RSM3 medium (10 mL) for 24 h, and AHG (10 mM) was added to each culture broth. All data shown are mean values from at least three replicate experiments. Error bars indicate standard deviations of the means (*n* = 3). Agarase activity **(A)** and cell growth **(B)** of the Δsco3485 mutant (□) and wild type *S. coelicolor* A3(2) (△) and the Δsco3485 mutant (◼) and wild type *S. coelicolor* A3(2) (▲) after feeding AHG.

The article "LacI-Family Transcriptional Regulator DagR Acts as a Repressor of the Agarolytic Pathway Genes in Streptomyces coelicolor A3(2)" was retracted in 2022. Reasons: fabricated or falsified data; fabricated or falsified images.

## Discussion

*S. coelicolor* A3(2) is known to have the ability to degrade agar, but its agarolytic pathway genes have not been widely studied. DagA, the first enzyme described in this pathway, is an endo-type β-agarase, and its expression is controlled by four different promoters at the transcriptional level; it is induced by agar but repressed by glucose (Buttner et al., 1987, 1988; Servin-Gonzalez et al., 1994). Recently, the transcriptomic analysis for carbon catabolite repression (CCR) has confirmed that most genes in the agarolytic pathway gene cluster, including the genes encoding for the three agarases, were repressed by glucose (Romero-Rodriguez et al., 2016, 2017). However, no changes in the expression of the only regulatory gene present in the cluster encoding a putative LacI-family transcriptional regulator (DagR) were detected (Romero-Rodriguez et al., 2016).

In this study, we demonstrated that the agarase activity of the *dagR* deletion mutant (Δsco3485) was significantly higher compared to that of the wild type strain (Figure 2). Furthermore, all the agarolytic pathway genes were significantly activated compared to other genes in the Δsco3485 mutant, suggesting that the enhanced agar degradation activity is essential for the derepression of DagR-mediated repression. Also, we confirmed that the DagR protein bound to the upstream regions of the three agarase genes (Figures 4, 5). Based on DNase 1 footprinting analysis, DagR-binding site was identified between positions -219 and –212 bp from the *dagA* translation start site with the consensus palindromic sequence AACCGGTT, which overlaps with the *dagA* transcription start site. Buttner et al. (1987) reported that the *dagA* gene was transcribed from four promoters located approximately 32, 77, 125, and 220 nt upstream of the coding sequence (Servin-Gonzalez et al., 1994). We subdivided the promoter region to investigate DagR-binding site (data not shown) and concluded that DagR bound to only one site of the upstream region of the *dagA* gene as shown in Figure 4. Thus, the DagR-binding site located at 219–212 nt upstream of the coding sequence showed a typical position for the repressor-binding site that interferes with the binding or the processing of RNA polymerase. The promoter region of *dagB* has two DagR-binding sites, one shared sequence with *dagA* promoter between –111 to –102 nt (aAACCGGTTt) and the other is located between –364 to –357 nt (GGACGTCC). Furthermore, the DagR-binding sequence in the *dagC* upstream region was different from that of *dagA* and *dagB*. This is in agreement with the binding motifs of the LacI-family transcriptional regulators, which contain inverted repeat sequences. It is possible that each binding sequence identified in this experiment could be related to the stability and specificity of DagR binding. The stability and specificity of transcriptional regulator binding are related to their binding affinities, which can be modulated to achieve desirable transcription activities (Du et al., 2019).

The article "LacI-Family Transcriptional Regulator DagR Acts as a Repressor of the Agarolytic Pathway Genes in Streptomyces coelicolor A3(2)" was retracted in 2022. Reasons: fabricated or falsified data; fabricated or falsified images.

The best understood transcriptional regulator, LacI repressor of *E. coli*, binds to *lac* operator and represses transcriptional initiation in the absence of a natural inducer, such as allolactose an analog of lactose created by a side reaction of β-galactosidase (Jobe and Bourgeois, 1972). It binds to a subunit of the tetrameric LacI repressor, which results in conformational changes and reduces the binding affinity of the LacI repressor to the *lac* operon (Weickert and Adhya, 1992; Daber et al., 2007). Interestingly, the binding affinity of DagR to target DNA sequences was reduced by a monosaccharide, AHG, but not by disaccharides, including neoagarobiose (Figure 7). Furthermore, we confirmed that the induction of agarase expression by AHG occurred only in the wild type strain (Figure 8). To the best of our knowledge, this is the first study to reveal that the only regulatory gene *dagR* present in the agarolytic pathway gene cluster of *S. coelicolor* A3(2) acts as a repressor for the three agarase genes, *dagA*, *dagB*, and *dagC*, and that AHG, one of the agar degradation products, inhibits the function of DagR.

In *Streptomyces* and other microorganisms, carbon source regulation is one of the most conserved mechanisms (Stulke and Hillen, 1999; Gorke and Stulke, 2008; Romero-Rodriguez et al., 2016). Although agarase overproduction by the Δsco3485 mutant in glucose-containing medium was less affected than in the wild type strain, CCR was similar to that in the wild type strain. This result is consistent with a previous study that the agarase activity of the cloned *dagA* gene in *Streptomyces lividans*, an evolutionary close strain lacking the DagR repressor, was reduced in the presence of glucose (Bibb et al., 1987; Park et al., 2014). Therefore, the regulatory mechanisms between CCR and DagR-specific repression are not independent and remain complex like CCR of other polysaccharides. More interrelated studies on the *dagA* gene regulation mechanism by DagR and CCR are required for further elucidation of DagR.

## Data Availability Statement

All datasets generated for this study are included in the article/Supplementary Material, further inquiries can be directed to the corresponding author/s.

The article "LacI-Family Transcriptional Regulator DagR Acts as a Repressor of the Agarolytic Pathway Genes in Streptomyces coelicolor A3(2)" was retracted in 2022. Reasons: fabricated or falsified data; fabricated or falsified images.

## Author Contributions

MT, SS, and C-RL performed the experimental work. C-RL, S-KH, and Y-SH drafted the manuscript. All authors were involved in designing, discussing, and interpreting the results of the experiments.

## Conflict of Interest

The authors declare that the research was conducted in the absence of any commercial or financial relationships that could be construed as a potential conflict of interest.

## References

[B1] BentleyS. D.ChaterK. F.Cerdeno-TarragaA. M.ChallisG. L.ThomsonN. R.JamesK. D. (2002). Complete genome sequence of the model actinomycete *Streptomyces coelicolor* A3(2). *Nature* 417 141–147. 10.1038/417141a 12000953

[B2] BibbM. J.JonesG. H.JosephR.ButtnerM. J.WardJ. M. (1987). The agarase gene (*dag A*) of *Streptomyces coelicolor* A3(2): affinity purification and characterization of the cloned gene product. *J. Gen. Microbiol.* 133 2089–2096. 10.1099/00221287-133-8-2089 3443853

[B3] ButtnerM. J.FearnleyI. M.BibbM. J. (1987). The agarase gene (*dagA*) of *Streptomyces coelicolor* A3(2): nucleotide sequence and transcriptional analysis. *Mol. Gen. Genet.* 209 101–109. 10.1007/BF00329843 17165236

[B4] ButtnerM. J.SmithA. M.BibbM. J. (1988). At least three different RNA polymerase holoenzymes direct transcription of the agarase gene (*dagA*) of *Streptomyces coelicolor* A3(2). *Cell* 52 599–607. 10.1016/0092-8674(88)90472-23342448

[B5] ChaterK. F.BiroS.LeeK. J.PalmerT.SchrempfH. (2010). The complex extracellular biology of *Streptomyces*. *FEMS Microbiol. Rev.* 34 171–198. 10.1111/j.1574-6976.2009.00206.x 20088961

[B6] ChiW. J.ChangY. K.HongS. K. (2012). Agar degradation by microorganisms and agar-degrading enzymes. *Appl. Microbiol. Biotechnol.* 94 917–930. 10.1007/s00253-012-4023-2 22526785

[B7] CobbR. E.WangY.ZhaoH. (2015). High-efficiency multiplex genome editing of *Streptomyces* species using an engineered CRISPR/Cas system. *ACS Synth. Biol.* 4 723–728. 10.1021/sb500351f 25458909PMC4459934

[B8] DaberR.StayrookS.RosenbergA.LewisM. (2007). Structural analysis of lac repressor bound to allosteric effectors. *J. Mol. Biol.* 370 609–619. 10.1016/j.jmb.2007.04.028 17543986PMC2715899

[B9] DuM.KodnerS.BaiL. (2019). Enhancement of LacI binding *in vivo*. *Nucleic Acids Res.* 47 9609–9618. 10.1093/nar/gkz698 31396617PMC6765135

[B10] GorkeB.StulkeJ. (2008). Carbon catabolite repression in bacteria: many ways to make the most out of nutrients. *Nat. Rev. Microbiol.* 6 613–624. 10.1038/nrmicro1932 18628769

[B11] HsiaoN. H.KirbyR. (2008). Comparative genomics of *Streptomyces avermitilis*, *Streptomyces cattleya*, *Streptomyces maritimus* and *Kitasatospora aureofaciens* using a *Streptomyces coelicolor* microarray system. *Antonie Van Leeuwenhoek* 93 1–25. 10.1007/s10482-007-9175-1 17588127PMC2140096

The article "LacI-Family Transcriptional Regulator DagR Acts as a Repressor of the Agarolytic Pathway Genes in Streptomyces coelicolor A3(2)" was retracted in 2022. Reasons: fabricated or falsified data; fabricated or falsified images.

[B12] JobeA.BourgeoisS. (1972). The *lac* repressor-operator interaction. VII. A repressor with unique binding properties: the X86 repressor. *J. Mol. Biol.* 72 139–152. 10.1016/0022-2836(72)90075-74567399

[B13] KendallK.CullumJ. (1984). Cloning and expression of an extracellular-agarase from *Streptomyces coelicolor* A3(2) in *Streptomyces lividans* 66. *Gene* 29 315–321. 10.1016/0378-1119(84)90060-x6489757

[B14] KieserT.BibbM. J.ButtnerM. J.ChaterK. F.HopwoodD. A. (2000). *Practical Streptomyces* genetics. Norwich: John Innes Foundation.

[B15] KimD. W.HeskethA.KimE. S.SongJ. Y.LeeD. H.KimI. S. (2008). Complex extracellular interactions of proteases and a protease inhibitor influence multicellular development of *Streptomyces coelicolor*. *Mol. Microbiol.* 70 1180–1193. 10.1111/j.1365-2958.2008.06471.x 18976279

[B16] LewisM. (2005). The *lac* repressor. *C. R. Biol.* 328 521–548. 10.1016/j.crvi.2005.04.004 15950160

[B17] NguyenC. C.SaierM. H.Jr. (1995). Phylogenetic, structural and functional analyses of the LacI-GalR family of bacterial transcription factors. *FEBS Lett.* 377 98–102. 10.1016/0014-5793(95)01344-x8543068

[B18] ParkJ.HongS. K.ChangY. K. (2014). Production of DagA, a beta-agarase, by *Streptomyces lividans* in glucose medium or mixed-sugar medium simulating microalgae hydrolysate. *J. Microbiol. Biotechnol.* 24 1622–1628. 10.4014/jmb.1405.05019 25085567

[B19] Perez-RuedaE.Collado-VidesJ. (2000). The repertoire of DNA-binding transcriptional regulators in *Escherichia coli* K-12. *Nucleic Acids Res.* 28 1838–1847. 10.1093/nar/28.8.1838 10734204PMC102813

[B20] RavcheevD. A.KhoroshkinM. S.LaikovaO. N.TsoyO. V.SernovaN. V.PetrovaS. A. (2014). Comparative genomics and evolution of regulons of the LacI-family transcription factors. *Front. Microbiol.* 5:294. 10.3389/fmicb.2014.00294 24966856PMC4052901

[B21] Romero-RodriguezA.RochaD.Ruiz-VillafanB.Guzman-TrampeS.Maldonado-CarmonaN.Vazquez-HernandezM. (2017). Carbon catabolite regulation in *Streptomyces*: new insights and lessons learned. *World J. Microbiol. Biotechnol.* 33:162. 10.1007/s11274-017-2328-0 28770367

[B22] Romero-RodriguezA.RochaD.Ruiz-VillafanB.TierrafriaV.Rodriguez-SanojaR.Segura-GonzalezD. (2016). Transcriptomic analysis of a classical model of carbon catabolite regulation in *Streptomyces coelicolor*. *BMC Microbiol.* 16:77. 10.1186/s12866-016-0690-y 27121083PMC4848846

[B23] SambrookJ.FritschE. F.ManiatisT. (1989). *Molecular Cloning: A Laboratory Manual*, 2nd Edn. Cold Spring Harbor, NY: Cold Spring Harbor Laboratory.

The article "LacI-Family Transcriptional Regulator DagR Acts as a Repressor of the Agarolytic Pathway Genes in Streptomyces coelicolor A3(2)" was retracted in 2022. Reasons: fabricated or falsified data; fabricated or falsified images.

[B24] Servin-GonzalezL.JensenM. R.WhiteJ.BibbM. (1994). Transcriptional regulation of the four promoters of the agarase gene (*dagA*) of *Streptomyces coelicolor* A3(2). *Microbiology* 140 2555–2565. 10.1099/00221287-140-10-2555 7528081

[B25] StulkeJ.HillenW. (1999). Carbon catabolite repression in bacteria. *Curr. Opin. Microbiol.* 2 195–201. 10.1016/S1369-5274(99)80034-410322165

[B26] TemuujinU.ChiW. J.ChangY. K.HongS. K. (2012). Identification and biochemical characterization of Sco3487 from *Streptomyces coelicolor* A3(2), an exo- and endo-type beta-agarase-producing neoagarobiose. *J. Bacteriol.* 194 142–149. 10.1128/JB.05978-11 22020647PMC3256618

[B27] TemuujinU.ChiW. J.LeeS. Y.ChangY. K.HongS. K. (2011). Overexpression and biochemical characterization of DagA from *Streptomyces coelicolor* A3(2): an endo-type beta-agarase producing neoagarotetraose and neoagarohexaose. *Appl. Microbiol. Biotechnol.* 92 749–759. 10.1007/s00253-011-3347-7 21655986

[B28] WeickertM. J.AdhyaS. (1992). A family of bacterial regulators homologous to Gal and Lac repressors. *J. Biol. Chem.* 267 15869–15874.1639817

[B29] YindeeyoungyeonW.SchellM. A. (2000). Footprinting with an automated capillary DNA sequencer. *Biotechniques* 29, 1034–1041. 10.2144/00295st05 11084866

